# Identification of a 5-Nutrient Stress-Sensitive Gene Signature to Predict Survival for Colorectal Cancer

**DOI:** 10.1155/2022/2587120

**Published:** 2022-04-18

**Authors:** Jingjie Xiong, Subing Xiong, Xi Feng, Huaming Zhang, Qisheng Su

**Affiliations:** ^1^Department of Cardiovascular Medicine, Liyuan Hospital, Tongji Medical College of Huazhong University of Science and Technology, Wuhan, Hubei 430071, China; ^2^Department of Gastroenterology, Zhijiang People's Hospital, Yichang 443000, China; ^3^Clinical Cardiovascular Center, Liyuan Hospital, Tongji Medical College, Huazhong University of Science and Technology, Wuhan, 430071 Hubei, China; ^4^Department of Clinical Laboratory, First Affiliated Hospital of Guangxi Medical University, Nanning, 530021 Guangxi, China

## Abstract

**Background:**

The high heterogeneity and the complexity of the tumor microenvironment of colorectal cancer (CRC) have enhanced the difficulty of prognosis prediction based on conventional clinical indicators. Recent studies revealed that tumor cells could overcome various nutritional deficiencies by gene regulation and metabolic remodeling. However, whether differentially expressed genes (DEGs) in CRC cells under kinds of nutrient deficiency could be used to predict prognosis remained unveiled.

**Methods:**

Three datasets (GSE70976, GSE13548, and GSE116087), in which colon cancer cells were, respectively, cultured in serum-free, glucose-free, or glutamine-free medium, were included to delineate the profiles of gene expression by nutrient stress. DEGs were figured out in three datasets, and gene functional analysis was performed. Survival analyses and Cox proportional hazards model were then used to identify nutrient stress sensitive genes in CRC datasets (GSE39582 and TCGA COAD). Then, a 5-gene signature was constructed and the risk scores were also calculated. Survival analyses, cox analyses, and nomogram were applied to predict the prognosis of patients with colorectal cancer. The effectiveness of the risk model was also tested.

**Results:**

A total of 48 genes were found to be dysregulated in serum, glucose, or glutamine-deprived CRC cells, which were mainly enriched in cell cycle and endoplasmic reticulum stress pathways. After further analyses, 5 genes, MCM5, MCM6, CDCA2, GINS2, and SPC25, were identified to be differentially expressed in CRC and be related to prognosis of in CRC datasets. We used the above nutrient stress-sensitive genes to construct a risk scoring model. CRC samples in the datasets were divided into low-risk and high-risk groups. Data showed that higher risk scores were associated with better outcomes and risk scores decreased significantly with tumor procession. Moreover, the risk score could be used to predict the probability of survival based on nomogram.

**Conclusions:**

The 5-nutrient stress-sensitive gene signature could act as an independent biomarker for survival prediction of CRC patients.

## 1. Introduction

Colorectal cancer (CRC) is one of the most common cancers worldwide and is the second most common cause of cancer death in the United States [1]. Increases in treatment options such as endoscopy and surgical resection, reduced preoperative radiotherapy and systemic therapy, targeted therapy, and immunotherapy have doubled the overall survival rate for patients with advanced CRC to 3 years [2], but the 5-year survival rate remains unsatisfactory [3]. Current prognostic models based on clinical predictors such as age, sex, and tumor lymph node metastasis (TNM) stage are still the gold standard for predicting prognosis in patients with CRC [4]. Though the treatment strategies and prognosis of patients have been greatly improved, drug resistance and insensitivity were still the unsolved problems. In addition, due to the high heterogeneity of colorectal cancer and the increasing complexity of the tumor microenvironment with the development of the disease, the prognosis based on conventional clinical indicators is not very accurate. Therefore, the establishment of new predictive features is crucial for the prediction of survival and drug design in patients with colorectal cancer.

It is known that cancer cells are often exposed to nutrient- and oxygen-deprived microenvironment due to poor blood vessel formation in developing tumor masses [5]. Tumor cells supported their survival and proliferation under these conditions through their metabolic plasticity. In cancer cells, glutamine was consumed voraciously, both for energy production and as a source of carbon and nitrogen for biomass accumulation [6]. Several studies have shown that cancer cells relied on the tumor suppressor p53-induced aspartate/glutamate transporter SLC1A3 or asparagine for cell survival after glutamine deficiency [7, 8]. Due to the high metabolic activity of tumor cells, the concentration of glucose as the main nutrient in tumor was much lower than that in normal tissues. Oxidative phosphorylation of mitochondria (OXPHOS) was the main pathway required for optimal proliferation of tumor cells under low-glucose conditions [9]. As tumors grow, tumor cells were often exposed to an anoxic environment, and they activated the transcription of many genes through overexpression of hypoxia-inducible factor 1 (HIF-1), which encoded proteins involved in angiogenesis, glucose metabolism, cell proliferation/survival, and invasion/metastasis [10]. From the above published work, we could see that cancer cells overcame various nutritional deficiencies through gene regulation and metabolic remodeling. Understanding these processes was crucial to develop new drugs or predict patient outcomes.

As a result, it has been critical to identify and enhance the characteristics that define patient prognosis in the early stages of the disease up to this point. On the other hand, the availability of noninvasive, cost-effective, and highly accurate biomarkers is critical for increasing patient enrollment in inexpensive screening programs and facilitating the diagnosis of CRCs in their early stages. In comparison, recent publications have demonstrated that noninvasive screening procedures such as cell-free circulating biomarkers are acceptable and possible, owing to the rapid advancement of high-throughput molecular technology over the last decade. A precise and robust gene signature can significantly aid in the clinical identification of disease [11]. Bioinformatics methods have been widely used to analyze high-throughput sequencing data and microarray data for the prediction of disease-related genes, such as renal cell carcinoma [12], triple-negative breast cancer [13], and colorectal cancer [14]. However, few of these studies examined the effect of nutritional deficiency in the tumor microenvironment on tumor prognosis, which was very important in tumor progression. We investigated the expression of differentially expressed genes in colorectal cancer cells under nutritional shortage using bioinformatics in this study. Five genes, MCM5, MCM6, CDCA2, GINS2, and SPC25, were shown to be differentially expressed in CRC and to be associated to CRC patients' prognosis in the datasets after gene ontology (GO) analysis and survival studies. The risk scores were then determined after constructing a 5-gene signature. Then, to forecast the prognosis of colorectal cancer patients and verify the performance of the risk model, survival analyses, cox analyses, and nomograms were used [15].

## 2. Methods

### 2.1. Data Preparing

First of all, a flow chart was shown to introduce this study design (Figure 1). By searching the key words “((starvation) OR (deprivation)) AND colorectal cancer” in the Gene Expression Omnibus (GEO) database (http://www.ncbi.nlm.nih.gov/geo/), three datasets (GSE70976, GSE13548, and GSE116087) were chosen for subsequent analysis. mRNA expression profiles from two groups that colorectal cancer cell line LoVo was cultured in normal or serum-free condition for 96 hours were extracted from GSE70976. Similarly, data that colorectal cancer cell line HT29 was cultured with normal or glucose-free medium for 18 hours was extracted from GSE13548. Transcription data via high throughput RNA sequencing in colorectal cancer cell line HCT116 grown in complete medium or in glutamine-free medium for 48 hours was downloaded from GSE116087. For signature identification, RNA sequencing data from GSE38592 consisting of 566 CRC and 19 normal samples was obtained, and 556 of which were finally selected as the training set after excluding normal samples and samples without key clinical features. Meanwhile, GDC TCGA Colon Cancer (COAD) cohort consisting of 512 samples was obtained from the Genomic Data Commons (GDC) Data Portal (https://portal.gdc.cancer.gov/). Normal samples, repeated samples, and samples without key clinical features were excluded for further analyses. After procession, there were 433 patients in GDC TCGA COAD project included as the test set.

### 2.2. Differentially Expressed Gene (DEG) Screening

The “limma” R package was utilized to calculate DEGs in GSE70976, GSE13548, and GSE116087 [16]. Adjust *P* value < 0.05 and |log_2_FC| > 1 were chosen to distinguish significant DEGs. Then, the overlapped gene list was acquired among the above three studies.

### 2.3. Functional Enrichment Analysis

To further explore the function of the overlapped gene, genes were exported and “clusterProfiler” R package was used to perform gene ontology (GO) analysis. “ggplot2” R package was used to present the first six enrichments of GO analysis. Moreover, genes were output to construct a protein-protein interaction (PPI) network by Cytoscape.

### 2.4. Survival Analysis and Statistical Analysis

Univariate and multivariate cox proportional hazards model and survival analyses were performed by the “survival” R package in combination with log-rank test to assess the differences. Two-tailed Student's *t*-test was used to compare two groups with normally distributed variables, and one-way analysis of variance was used for mutigroup comparison. *P* < 0.05 was considered statistically significant.

### 2.5. Predictive Gene Signature Construction

The risk score of each sample was calculated by the formula risk score = exp_mRNA1_∗*β*_mRNA1_ + exp_mRNA2_∗*β*_mRNA2_ + ⋯+exp_mRNAn_∗*β*_mRNAn_. “exp” represents the mRNA expression, and “*β*” is referred to as the mRNA coefficient derived from the univariate cox regression analysis.

## 3. Results

### 3.1. DEG Screening

To delineate the profile of gene expression by nutrient stress, we included three datasets (GSE70976, GSE13548, and GSE116087), in which colon cancer cells were cultured in serum-free, glucose-free, or glutamine-free medium, respectively. In GSE70976 with serum deprivation, 5091 differentially expressed mRNAs were obtained under the criteria of adjust *P* value < 0.05 and |log · FC| > 1, including 3146 upregulated mRNAs and 1945 downregulated mRNAs. With the same criteria, only 268 DEGs were obtained in GSE13548, while 126 were upregulated and 142 downregulated. In GSE116087 with glutamine starvation, there were 1258 DEGs with 778 upregulated and 481 downregulated. Venn diagram showed that a total of 48 genes were significantly influenced by three kinds of nutrient deprivation conditions in colon cancer cells (Figure 2(a)). To further explore the characteristics of the above 48 genes, GO analysis was performed. Data showed that endoplasmic reticulum (ER) stress-related pathways and cell cycle related pathways were significantly enriched in these genes (Figure 2(b)). PPI network divided the 48 genes into two separate subnetworks. Genes in one subnetwork were all cell cycle related while those in the other were ER stress related. More interestingly, cell cycle-related genes were downregulated under nutrient deprivation when ER stress-related genes were upregulated (Figure 2(c)). The above data demonstrated that nutrient stress could induce the expression alterations of cell cycle and ER stress-related genes.

### 3.2. Differentially Expression Identification of Nutrient Stress-Sensitive Genes in CRC

Then, an online Gene Expression Profiling Interactive Analysis (GEPIA) database (http://gepia.cancer-pku.cn/) was used to identify the differential mRNA expression of the 48 genes, which actively responded to nutrient stress, between cancers and normal tissues. In Figure 3(a), data showed that the mRNA expression levels of MCM5, MCM6, CDCA2, GINS2, and SPC25 (*P* < 0.05) were upregulated in CRC tumor tissues when compared with those in nontumor tissues. Immunohistochemistry staining obtained from the Human Protein Atlas database revealed strong increase in the protein levels of the above genes in CRC tumor tissues, compared with normal colon tissues (Figure 3(b)). Furthermore, the expression of MCM5, MCM6, and CDCA2 (*P* < 0.05) was significantly decreased with the progression of CRC while GINS2 and SPC25 (*P* > 0.05) had no significance (Figure 3(c)).

### 3.3. Expression Pattern and Survival Analyses of the 5 Nutrient Stress-Sensitive Genes in CRC Datasets

Next, we used the training set (GSE39582) and the test set (TCGA COAD) to verify the expression pattern of the 5 nutrient stress-sensitive genes. As shown in Figure 4, in the training set, we found that the expression of MCM5, CDCA2, GINS2, and SPC25 (*P* < 0.05 or *P* < 0.001) was significantly decreased with the progression of CRC while MCM6 (*P* > 0.05) had no significance (Figure 4(a)). But in the test set, the expression of MCM5, MCM6, and CDCA2 (*P* <0.05 or *P* < 0.001) was negatively correlated with CRC stage, while the expression of GINS2 and SPC25 (*P* > 0.05) was not significantly correlated with tumor stage (Figure 4(b)). We then investigated the relationship between the 5 genes (MCM5, MCM6, CDCA2, GINS2, and SPC25) and overall survival (OS) of patients in both the training set and test set. In the training set, data showed that low expression of these five genes was associated with poor prognosis (*P* < 0.001, Figure 4(c)), while in the test set, result indicated that low expression of MCM6, CDCA2, and GINS2 (*P* < 0.05) was related to worse outcome while MCM5 and SPC25 (*P* > 0.05) were not (Figure 4(d)).

### 3.4. Construction of a 5-Gene Signature Risk Scoring System

The above data showed that the single-nutrient stress-sensitive gene could not well predict prognosis of CRC patients; therefore, we applied a risk scoring algorithm to construct a 5-gene signature for evaluating the prognosis of patients with CRC. According to the results of univariate Cox regression analysis in the training set (Table S1), the risk score was determined for each sample based on the mRNA expression and coefficient of the 5 nutrient stress-sensitive genes. Then, by “Survminer” package, we calculated the cutpoint in both the training set (10.81) and test set (20.86), which divided CRC samples into two groups, with those greater than the cutpoint being classified as the high score group and those less than cutpoint being classified as the low score group (Figures 5(a) and 5(c)). In addition, we included clinical factors in this study, and further multivariate Cox analysis found that age, stage, and risk score could be used as independent prognostic factors to evaluate patients' survival time in both the training set and test set (Figures 5(a) and 5(c)). The result showed that patient had a low age and a low tumor stage would have a better prognostic while with a low risk score would have a worse outcome.

### 3.5. Prognostic Roles of the 5-Gene Signature Risk Scoring Systems

We analyzed the relationship between risk score and tumor stage in both the training set and test set (Figures 6(a) and 6(c)); the results showed that the risk score decreased with the progression of tumor stage (*P* < 0.001). We also examined the relationship between risk scores and the OS of patients and found that patient with a high risk score would have a better prognostic in both sets (Figure 6(b): *P* = 0.0003; Figure 6(d): *P* = 0.0024). In addition, the relationship between the risk scoring model and OS was evaluated using a survival probability prediction model based on the nomogram (Figures 7(a) and 7(c)). We assessed 5- and 10- year survival at each time point in the training and test sets after the overall scores for risk score, tumor stage, and age were positioned on the total score scale. The nomogram model showed that patients in the high-risk score group showed a better probability of survival. In addition, we found that the 5-year and 10-year survival predicted by the risk score model was very close to the actual observed survival rates from the training and test sets, respectively (Figures 7(b) and 7(d)), indicating the high accuracy of the method.

## 4. Discussion

In the process of tumor formation, tumor cells usually have to survive in an environment lacking nutrition and oxygen. Understanding this process is important for us to predict the prognosis of patients. Therefore, in this study, we identified a 5-gene signature (MCM5, MCM6, CDCA2, GINS2, and SPC25) for CRC after analyzing the gene expression profiles of colorectal cancer cells in the absence of nutrients. Then, a novel risk score model to predict the OS of CRC patients was constructed based on the 5-gene signature. Multivariate Cox analysis found that risk score could be used as an independent prognostic factor to evaluate patients' survival time in both the training set and test set. We also found that the risk score decreased with tumor progression. Finally, the nomogram based on risk score, tumor stage, and age was established to predict prognosis of CRC patients.

DNA replication is a hot topic in the study of tumorigenesis and development, in which microchromosome maintenance family (MCM) plays a key role in replication. The MCM family has many homologues and performs different functions. They were mostly overexpressed in tumors and are associated with poor prognosis [17]. Minichromosome maintenance deficient 5 (MCM5) belongs to the microchromosome maintenance complex, which drives the formation of the prereplication complex during the first critical event of the G1 phase and is essential for cell proliferation [18]. MCM5 was overexpressed in many cancers, such as urothelial carcinoma [19], bladder cancer [20], and renal cell carcinoma [21], and was associated with poor prognosis. Our data showed that MCM5 was upregulated in CRC. However, our data further showed that high expression of MCM5 was associated with better outcome, which was not consistent with its role in other cancers. In anaplastic thyroid cancer (ATC), MCM5 directly bound to the bromine domain and terminal (BET) protein BRD4 to regulate cell proliferation and may be a new target for ATC therapy [22]. Overexpression of MCM5 was associated with poorer tumor staging in laryngeal squamous cell cancer [23], contrary to the conclusion of our study that MCM5 expression gradually decreased with CRC progression. MCM5 was usually overexpressed in colorectal cancer cells [24], but more researches were needed to explore the specific mechanisms of MCM5 in colorectal cancer.

Minichromosome maintenance deficient 6 (MCM6) also belongs to the microchromosome maintenance family, and its function is similar to that of MCM5 [25]. MCM6 was highly expressed in tumors such as liver cancer [26], breast cancer [27], and glioma [28] and was associated with poor prognosis. In liver cancer, MCM6 promoted cancer metastasis through the MEK/ERK pathway [29]. In colorectal cancer, MCM6 expression levels would negatively correlate with the tumor stage and its high expression level was associated with a favourable outcome [30], which was consistent with our results.

Cell division cycle-associated 2 (CDCA2) was one of the 5 nutrient stress-sensitive genes in our study. CDCA2 is a nucleoprotein that specifically binds to protein phosphatase 1*γ* (PP1*γ*) and regulates DNA damage responses during the cell cycle [31, 32]. CDCA2 forms a complex with PP1*γ* to preserve chromosome structure during mitosis, and CDCA2 promotes dephosphorylation of major mitotic histone H3 [33]. CDCA2 was overexpressed in many cancers, such as lung cancer [34], invasive neuroblastoma [35], and oral squamous cell carcinoma [36], and was associated with poor prognosis. A study has shown that CDCA2 was also overexpressed in colorectal cancer and promoted CRC cell proliferation and tumorigenesis through overexpression activation of the PI3K/Akt pathway [37]. This contradicted our conclusion that high expression of CDCA2 was associated with better prognosis and that its expression decreased with tumor progression. Therefore, more studies were needed to clarify the role of CDCA2 in CRC.

GINS complex subunit 2 (GINS2) belongs to the GINS complex family and plays a critical role in the initiation of DNA replication and the cell cycle. The GINS family correctly establishes and maintains DNA replication forks through stable interactions with the MCM 2-7 complex and CDC45 [38]. Several studies have shown that GINS2 was highly expressed in many tumors. One study showed that GINS2, which was usually overexpressed in triple-negative breast cancer cells, could enhance tumor proliferation by promoting cell cycle progression, and its abundance was associated with tumor progression in patients [39]. Another study has shown that GINS2 was highly expressed in early cervical cancer and was associated with poor prognosis. In addition, inhibition of GINS2 could inhibit the proliferation, tumorigenicity, and invasion of cervical cancer cells [40]. There have been no reports of GINS2 in CRC, and our study showed that high GINS2 expression level was associated with better prognosis, which was contrary to the conclusions obtained in other tumors, so a large number of studies were needed to confirm our conclusions.

Spindle pole body component 25 (SPC25) is a component of the nuclear division cycle 80 (Ndc80) complex, which is essential for chromosome separation [41]. Some studies have found that dysregulation of SPC25 was associated with oncogenic processes and malignant phenotypes of some cancers. High expression of SPC25 has been found to be associated with poorer prognosis in breast cancer. Another study has shown that SPC25 upregulation increased cancer stem cell characterization in non-small-cell lung adenocarcinoma cells and was associated with poorer prognosis. In one article, SPC25 was upregulated in colorectal cancer which was consistent with our findings. However, our data show that high expression of SPC25 was associated with better prognosis, which was inconsistent with the results observed in other tumors, and further investigation was needed.

As a new diagnostic test for determining the likelihood of recurrence in stage CRC patients after surgical resection, since 2010, the Oncotype DX colon cancer test has been commercially accessible in the United States and across the world. The findings revealed that this five-gene signature might be a valuable tool for the management of patients with colorectal cancer. Due to the retrospective nature of our work, its dependability should be confirmed in a large prospective investigation [42].

Our research is novel in the following ways. To begin, a subsequent multivariate Cox analysis revealed that age, stage, and risk score were associated with favourable prognostic ability. Second, our work is a comprehensive assessment of prognostic gene signatures in colorectal cancer (CRC). Thirdly, our study offers a number of strengths in terms of design and analytical approaches. The five-gene classifier was verified using independent in silico datasets and a clinical cohort from an independent community. Due to the fact that we established a “risk prediction model” based on our five-gene signature, the scores may be easily applied to independent prospective cohorts in the future [43].

As far as we know, our study was a pioneer work to reveal the relationship between the above 5 nutrient stress sensitive genes and OS in CRC. But the study still had many shortcomings. First of all, more datasets by nutrient deprivation in CRC were needed to validate the differential expression of the 5 genes. Then, our data showed that the 5 genes were all downregulated in nutrient-deprived CRC cells, but whether and how the absence of these genes contributed to the survival of CRC cells needed basic researches.

## 5. Conclusion

We constructed a new risk score model for predicting prognosis in patients with CRC based on the 5 nutrient stress sensitive genes. The model showed that CRC patients with higher risk scores were associated with better outcomes and that risk score decreased significantly with tumor staging. Finally, we established a nomogram based on risk score, tumor stage, and age to predict prognosis of CRC patients.

## Figures and Tables

**Figure 1:** A flow chart of the study.

**Figure 2:** DEGs and GO analysis of nutrient stress-sensitive genes. (a) Venn diagram showed the number of DEGs among three kinds of nutrient deprivation in CRC cells. (b) GO analysis results of the nutrient stress-sensitive genes. (c) PPI network of the nutrient stress-sensitive genes. DEGs: differentially expressed genes; GO: gene ontology; PPI: protein-protein interaction.

**Figure 3:** Expression identification of the 5 nutrient stress-sensitive genes in CRC. (a) mRNA expression levels of MCM5, MCM6, CDCA2, GINS2, and SPC25 in CRC tumor tissues and normal tissues. (b) Protein expression levels of MCM5, MCM6, CDCA2, GINS2, and SPC25 in CRC tumor tissues and normal tissues. (c) mRNA expression levels of MCM5, MCM6, CDCA2, GINS2, and SPC25 in different stages of CRC. ^∗^*P* < 0.05.

**Figure 4:** Expression levels and survival analyses of the 5 nutrient stress-sensitive genes in CRC datasets. (a, b) mRNA expression levels of MCM5, MCM6, CDCA2, GINS2, and SPC25 in different CRC stages of the GSE39582 dataset (a) and TCGA COAD dataset (b). (c, d) Survival analyses of MCM5, MCM6, CDCA2, GINS2, and SPC25 in the GSE39582 dataset (c) and TCGA COAD dataset (d).

**Figure 5:** A 5-gene signature risk scoring system construction. (a, c) Cutpoint calculation of the risk scores in the GSE39582 dataset (a) and TCGA COAD dataset (c). (b, d) Multivariate Cox analysis of the risk scores in the GSE39582 dataset (b) and TCGA COAD dataset (d).

**Figure 6:** Expression levels and survival analyses of the risk scores. (a, c) mRNA expression levels of the risk scores in the GSE39582 dataset (a) and TCGA COAD dataset (c). (b, d) Survival analyses of the risk scores in the GSE39582 dataset (b) and TCGA COAD dataset (d).

**Figure 7:** Nomogram model for prognosis prediction by the 5-nutrient stress-sensitive gene signature combined with clinical traits in CRC patients. (a, c) The nomogram model showed the survival probability in the GSE39582 dataset (a) and TCGA COAD dataset (c). (b, d) Calibration curve of the nomogram model. The *x*-axis represents the nomogram-predicted probability of overall survival, and the *y*-axis showed the actual survival probability.

## Data Availability

TCGA data were extracted from GDC data portal (https://portal.gdc.cancer.gov/). The GSE39582 gene expression profiles were downloaded from GEO (https://www.ncbi.nlm.nih.gov/geo).

## Abbreviations

CRC: Colorectal cancer
PPI: Protein-protein interaction
DEG: Differentially expressed gene
GO: Gene ontology
KEGG: Kyoto Encyclopedia of Genes and Genomes
OS: Overall survival
ER: Endoplasmic reticulum.

## Supplementary Materials

Supplementary 1 Table S1: gene symbols of the 48 nutrient stress-sensitive genes.

Supplementary 2 Table S2: univariate Cox regression analysis of the 5 genes.
